# A Cabled Acoustic Telemetry System for Detecting and Tracking Juvenile Salmon: Part 1. Engineering Design and Instrumentation

**DOI:** 10.3390/s110605645

**Published:** 2011-05-26

**Authors:** Mark A. Weiland, Z. Daniel Deng, Tom A. Seim, Brian L. LaMarche, Eric Y. Choi, Tao Fu, Thomas J. Carlson, Aaron I. Thronas, M. Brad Eppard

**Affiliations:** 1 Pacific Northwest National Laboratory, P.O. Box 999, Richland, WA 99332, USA; E-Mails: Thomas.Seim@pnl.gov (T.A.S.); brian.lamarche@pnl.gov (B.L.L.); eric.choi@pnl.gov (E.Y.C.); tao.fu@pnnl.gov (T.F.); thomas.carlson@pnl.gov (T.J.C.); aaron.thronas@pnnl.gov (A.I.T.); 2 U.S. Army Corps of Engineers, Portland District, P.O. Box 2946, Portland, OR 97208, USA; E-Mail: matthew.b.eppard@usace.army.mil

**Keywords:** acoustic telemetry, microtransmitter, juvenile salmon

## Abstract

In 2001 the U.S. Army Corps of Engineers, Portland District (OR, USA), started developing the Juvenile Salmon Acoustic Telemetry System, a nonproprietary sensing technology, to meet the needs for monitoring the survival of juvenile salmonids through eight large hydroelectric facilities within the Federal Columbia River Power System (FCRPS). Initial development focused on coded acoustic microtransmitters and autonomous receivers that could be deployed in open reaches of the river for detection of the juvenile salmonids implanted with microtransmitters as they passed the autonomous receiver arrays. In 2006, the Pacific Northwest National Laboratory began the development of an acoustic receiver system for deployment at hydropower facilities (cabled receiver) for detecting fish tagged with microtransmitters as well as tracking them in two or three dimensions for determining route of passage and behavior as the fish passed at the facility. The additional information on route of passage, combined with survival estimates, is used by the dam operators and managers to make structural and operational changes at the hydropower facilities to improve survival of fish as they pass the facilities through the FCRPS.

## 1. Introduction

Migrating fish may be injured or killed when they pass through hydroturbines and other passage routes at hydroelectric facilities [1–6]. In the Columbia and Snake River basins, several species of anadromous Pacific salmon are currently listed for protection under the Endangered Species Act of 1973 due to population declines. The 2008 Federal Columbia River Power System Biological Opinion (FCRPS BiOp; [7]) includes standards to be met to make hydroelectric facilities more fish-friendly through operational changes, improved hydroturbine design, and other structural or operational changes. Implementing and testing these changes require reliable estimates of behavior, timing, and survival of the juvenile salmonids as they migrate downstream through the FCRPS and into the Pacific Ocean [8–11].

The Juvenile Salmon Acoustic Telemetry System (JSATS) is a nonproprietary sensing technology developed by the U.S. Army Corps of Engineers (USACE), Portland District, for evaluating behavior and survival of juvenile salmonids migrating through the FCRPS. Receivers have been deployed at large hydroelectric dams, in free-flowing sections of the FCRPS, and in the estuary of the Columbia River [12]. The JSATS consists of acoustic microtransmitters; autonomous, cabled, or portable receivers with hydrophones; and data management and processing applications.

Self-contained autonomous receivers that detect, decode, and store decoded messages are typically deployed in areas within the Columbia River basin where a power source is not readily available and cable runs are not feasible [12,13]. General fisheries applications of JSATS and the autonomous receivers were reported in 2010 [12]. Portable receivers detect, decode, store, and display transmitted signals for in-laboratory transmitter testing and for displaying and entering transmitter codes at the time of tagging. A mobile receiver consisting of a single four-hydrophone cluster deployed from a mobile platform (e.g., a single boat) has been used to provide two-dimensional (2D) and three-dimensional (3D) position estimates on actively migrating tagged fish. Cabled receivers detect, decode, and store decoded messages, time of arrival (TOA), and message waveforms as received, on up to four hydrophones per four-channel receiver system. These receivers are typically located at large hydroelectric dams within the FCRPS and are used for estimating route and time of passage, including 2D and 3D position estimates for tagged fish. TOA information for valid detections on at least four hydrophones is required to solve for 3D position, and TOA information from at least three hydrophones is required to resolve for 2D position [14–21]. Cabled receivers are intended for deployment primarily at dams or other locations where cabled hydrophones can be deployed, electricity is available, equipment can be maintained without undue logistical complexity or cost, and immediate access to received transmitter messages is desirable. The cabled receivers also provide synchronization and high accuracy in the time of receipt of transmitter messages across an array of many hydrophones when required. In addition to fixed-location hydrophone arrays, cabled receivers also satisfy requirements for mobile arrays that may be deployed in fixed geometries from boats.

In this article, we describe in detail the engineering design and implementation of the current version of the JSATS cabled system. In Part 2 [22], 3D tracking and error analysis using JSATS cabled systems are presented and evaluated.

## 2. System Overview

A typical cabled JSATS system consists of acoustic microtransmitters, four hydrophones, four cables, a signal conditioning interface/amplifier, JSATS detector using digital signal processing (DSP) + field-programmable gate array (FPGA), a Global Positioning System (GPS) receiver, data acquisition computer, and decoder software (Figure 1).

The acoustic microtransmitter, surgically implanted in the fish [23,24], translates a programmed binary code into an acoustic message. The acoustic signal is transmitted through freshwater at approximately 1,500 m/s. When the study fish implanted with the microtransmitters travel within the detection range of the deployed receivers, the acoustic signals in the form of sound pressure levels are converted into a very low analog voltage by the piezoelectric sensors at the tip of the hydrophones [25,26]. The four hydrophones, deployed underwater in a known fixed geometry, have an internal preamplifier that amplifies the low analog voltage signal. These hydrophones are connected by cables to a signal conditioning interface. The pre-amplified analog signal is then transmitted to the signal conditioner for further amplifying and conditioning prior to being input to a DSP + FPGA card resident in the data acquisition computer for detection analysis. The signal conditioning interface and the JSATS detector using DSP + FPGA are both designed to simultaneously process the data from all four receiver hydrophones. The times of receipt of candidate encoded messages at hydrophones in a multisystem array are synchronized across the array to submicrosecond accuracy using GPS receivers (Meinberg GPS 170PCI, Meinberg Funkuhren GmbH & Co. KG, Bad Pymont, Germany).

*Detection* is the decision whether to collect a portion of the incoming signals. The process of detection analysis is described in detail in Section 3.4. The first step in detection is digitization of the received analog signal. Processing algorithms evaluate the stream of digital data to identify candidate microtransmitter messages. Portions of the signals entering the DSP + FPGA that do not pass candidate microtransmitter identification criteria are classified as noise and ignored. If criteria for a candidate microtransmitter message are met, the DSP grabs a high-resolution time stamp from the GPS clock that corresponds to the initial receipt of the candidate microtransmitter message. The data is now a digitized waveform represented as a series of short integers (16 bits) and a high-precision time stamp acquired from the GPS clock card. The digital candidate microtransmitter message waveform is sent to the data acquisition computer and saved to disk in a custom format called the binary waveform format. The structure for a candidate message waveform file contains a header and a data payload. The header describes the data payload and the instruments used to digitize the analog waveform (e.g., the analog-to-digital converter resolution or number of hydrophone data the file contains). The data payload is where the digitized signal is stored. A binary format is selected to save hard drive space.

Once stored as a binary file, the candidate message data is available for decoding. The decoding software reads the binary file and converts the data from short integer format into double floating-point format for better accuracy. The decoding software then processes the saved waveform file searching for valid microtransmitter messages. Each detected message is given a relative and absolute TOA. The relative TOA is the start of the decoded microtransmitter message time in microseconds relative to the start of the complete candidate message waveform file. The absolute TOA is the time of the start of the decoded microtransmitter message in seconds from the start of the day with microsecond fractional time information. The microtransmitter message decoding and TOA information are then sent to file (typically in a database) for further processing to provide the information required to meet study objectives.

## 3. Instrumentation

### 3.1. Acoustic Microtransmitters

Each microtransmitter, surgically implanted in study fish, transmits a unique binary code encoded using binary phase shift keying (BPSK) as a 416.7-kHz carrier waveform, ±0.5% (2.08 kHz). The source level of the current microtransmitter design is larger than +153 dB re 1 μPa @ 1 m. It has a maximum weight of 0.430 g in air. Its maximum dimensions are 6.00 mm wide, 4.10 mm thick, 12.00 mm long, and 0.300 mL in volume (Figure 2).

The code structure of the mictotransmitter includes a total of 31 bits, with 7 synchronization bits (Barker code 1110010 in bits or 72 in hexadecimal format), 16 ID bits (4 hexadecimal digits), and 8 cyclic redundancy check (CRC) bits (2 hexadecimal digits), resulting in the 65,536 possible unique identification codes. BPSK was chosen for encoding because of its excellent bit error rate performance in noisy environments. A bit change from 0 to 1 or 1 to 0 results in a phase change of 180 degrees in the carrier (no phase change occurs if the next bit is the same). Unlike an electrical signal, phase change requires several cycles when the piezoelectric transducer changes its phase of oscillation and a vibrating mass cannot instantly modify the phase of vibration. This is apparent in the waveform as a slight lengthening of the time between message bits as the new phase is achieved. The active element may also shorten (speed up) the time between bits as it changes phase, but this is much less common. During the phase change, the magnitude of oscillation decreases. The physical requirements for change in phase are evident in microtransmitter waveforms (Figure 3). Each transmitted bit requires 10 carrier cycles. The microtransmitters emit their unique 31-bit codes at a programmed interval, typically every 3, 5, or 10 s, depending on the study design, for 310 cycles at a carrier period of 2.4 μs, resulting in a signal length of 744 μs and an acoustic length of approximately 1.1 m at 20 °C.

### 3.2. JSATS Cabled Hydrophone

The function of the hydrophones is to convert incident acoustic pressure to an analog voltage signal and to amplify the signal for transmission. Requirements for accuracy in the position estimates of the hydrophones can vary considerably, depending upon the measurement objective driving a deployment. A number of systems [Figure 4(a)] may be installed to create an array consisting of a large number of hydrophones. All hydrophones are synchronized to the universal GPS clock using a GPS card, resulting in detection time accuracy on a single system (an array of four hydrophones) to 250 ns and across multiple systems to 500 ns.

The JSATS cabled hydrophones (Model 2008, Sonic Concepts Inc., Seattle, WA, USA) are cylindrical and have a weight of 800 g in air with acoustic element on a reinforced stalk [Figure 4(b)]. The acoustic element potting material has acoustic impedance nearly that of freshwater and is resistant to fresh- and seawater; the shoulder between the element stalk and amplifier housing is shaped to reflect sound away from the acoustic element. JSATS hydrophones are narrow-band (±42 kHz to 3 dB points) with a center frequency of 416.7 kHz and may have any directivity between omnidirectional to very directional, depending on applications. The hydrophones have an operational depth of 100 m, and the built-in low-noise pre-amplifier allows an adjustable gain within the range of 26 to 55 dB. The hydrophones have a sensitivity of −180 ±2 dB re 1 V/μPa at beam center with 100 ohm differential output termination.

The JSATS underwater cables for the hydrophones are mechanically and electrically terminated with underwater terminations at the ends that connect to a hydrophone and by “dry” terminations at the ends that connect to the signal conditioning interface. The cables may or may not have a strength member integral to their construction.

### 3.3. JSATS Signal Conditioner

The four hydrophones in a JSATS cabled system are connected by cables to a four-channel JSATS signal conditioner (Precision Acoustic Systems, Seattle, WA, USA). The JSATS signal conditioner amplifies and conditions the analog signals prior to signal detection analysis. Detailed specifications of the JSATS signal conditioner are as follows:

1. A power supply with +6 and −6 V is required.
2. Four independent receiver channels (with common power supply).
3. Input self-noise must be less than 3 nV/SqrtHz (for 90-ohm source).
4. MS3102A14S-6S hydrophone signal-input/pre-amp power connector on the rear panel (signal−/−6 V > B&C, signal+/+6 V > E&F, signal common > A&D).
5. 3-wire (2008 model) or 6-wire (2010 model) common-mode choke with a common-mode impedance of more than 35 K-ohm from 342 to 492 kHz for all inputs.
6. Differential input signal impedance at 416.667 kHz of 85 to 95 ohm.
7. Individual gain control inputs for each channel (female BNC on front panel) with a scale factor of 20 dB/V, an input resistance > 100 K-ohm, and a common mode range of −2.0 to +0.5 V. The control voltage is typically 0 to 4 V for an 80-dB gain control range.
8. Maximum receiver gain at 0 V is less than 16 dB when the gain-control voltage is at 0 V.
9. Three-pole Bessel filter or better with a 150-kHz bandwidth centered at 416.667 kHz and matched to within 3% in both amplitude and phase.
10. Each input channel has a BNC connector for signal outputs on the front panel.
11. Each receiver channel must be equalized within 0.5 dB over a 60-dB gain-control range.
12. A power entry module on the front panel with fuse holder and on/off switch (115 V AC) is required.
13. The instrument case must be a standard 17-in. rack mount case with front rack-mount handles.

### 3.4. Detector

A DSP + FPGA card (digital signal processor TMS320C6713 and field programmable gate array Xilinx XC3S1000, Innovative P25M; Innovative Integration, Simi Valley, CA, USA) resident in the data acquisition computer is used for digitization and detection analysis. Detection analysis begins after the analog signal out of the quad-amplifier has been digitized and error-corrected by the DSP + FPGA card. The digital signal is processed to determine if there is a candidate transmitter message. Candidate messages are identified by performing a cross-correlation of the received acoustic signals with a known square function that is the same length as a transmitter message, which is 1,860 samples long. It is equivalent to computing windowed energy with a window size of 1,860 samples. When a candidate message is present, the cross-correlation peaks at the beginning of the candidate message.

The coding architecture for the detector consists of three components. The first component deals with the logic in the FPGA and is written in VHDL (VHSIC [Very High Speed Integrated Circuits] Hardware Description Language) and coded using the Xilinx ISE (Integrated Software Environment). The second component deals with the DSP and is coded in C using the Code Composer Studio IDE (Integrated Development Environment). The third component is the user interface incorporated with the host program to send and receive information from the DSP + FPGA PCI card and the user interface is coded in C++ using Visual Studio.

Framework Logic is provided for the P25M board by Innovative Integration as a VHDL-based project in the Xilinx ISE environment. This framework provides an environment that connects the onboard analog-to-digital converter (ADC) and digital-to-analog converter (DAC) with the DSP. The framework logic allows for control of the ADC and DAC settings and also provides captured data to the DSP logic. Through the DSP logic, the user is able to process the data and have it transferred to the host computer. The cross-correlation calculations on the ADC data are handled in the FPGA logic using two multipliers—a FIFO (first-in first-out) and an accumulator. The raw data and cross-correlation data are then passed along to the DSP to identify the packets of data to save to a data file. The DSP code allows for the simple passing of ADC data from the FPGA to the host computer. Each packet of data processed by the DSP is 8,192 samples of raw data. Two thresholds are used for detection analysis. The first is a function of background noise, usually set 1.5 to 2 times the background noise. The second threshold is the number of samples above the first threshold with the cross-correlation values at these samples monotonically increasing. If these thresholds are met by the cross-correlation, then a candidate message is detected. To ensure the entire signal and any possible reflections are captured, one packet before this detection and three packets after this detection are sent over to the host PC to be saved, resulting in 40,980 samples or 16 ms in recording time per data file.

The host code is a modification of the original host code provided by Innovative Integration. This code had premade dynamic-link libraries (DLLs) that make it easy to interact with the installed PCI board containing the FPGA and DSP. This code has been modified to save the data from the ADC in customized file format. Other changes made to the host program are the ability for the user to choose the location to which the data should be saved and the base waveform file name. This code provides a simple interface for the user to interact with the DSP + FPGA board.

As an example, if we set the first threshold to twice that of background noise and the second threshold to 250, the correlation values corresponding to an impulse noise (Figure 5) are larger than the first threshold, but the number of samples above the first threshold with the correlation values monotonically increasing is only 152, smaller than the second threshold. As a result, this impulse noise does not pass the JSATS detector and will not be saved to the host computer. However, for another example, when a real JSATS acoustic signal passes along (Figure 3), the number of samples above the first threshold with the correlation values monotonically increasing is 1,820 and larger than the second threshold (Figure 6). Therefore, this packet is determined to be a JSATS signal by the detector, and one packet before this packet and three packets after this packet are sent over to the host PC for archiving. The analog voltage signal from the JSATS cabled hydrophone is digitally sampled at a frequency of 2.5 MHz. The high sampling frequency allows accurate representation of JSATS 416.7-kHz signals with at least six samples per signal cycle.

### 3.5. Decoder

The BPSK decoder was separate from the detector and host environment. It was implemented and evaluated in MathWorks MATLAB 7.0 before it was translated into C++ for optimization as a standalone utility. The major steps required to successfully decode a JSATS acoustic microtransmitter message are (1) estimate the most likely message locations and compute the corresponding phase angles; (2) decode the candidate messages and validate the messages; (3) compute the time difference of arrivals between different hydrophones for selected messages, given the time of arrival of each decoded message at the hydrophones.

The detailed steps for estimating the most likely message locations and computing the corresponding phase angles are as follows:

1. Locate all carrier peaks and their locations in the time-domain waveform. Insert or delete peaks as necessary to maintain cycle accuracy (*i.e.*, one peak for each of the 6-sample cycles).
2. Compute signal energy using the peaks and correlate the signal energy with one message size (310 cycles) to obtain total energy within one message.
3. Search for predefined number of energy peaks (usually set to 5) from the energy obtained from step 2.
4. Locate the start of signals corresponding to the energy peaks. These signal starts are the most likely message locations.
5. Compute the signal-to-noise ratio (SNR) of the time-domain waveform around each of the most likely message locations.
6. Screen signals above the predefined minimum SNR.
7. Estimate frequency and phase of signal using statistical properties of the phase distribution.
8. Convert the time-domain waveform to phase data.
9. Convert the phase data into bipolar bits by comparing the phase data to a decision threshold (each bit represents one carrier cycle).

The detailed steps for decoding the messages after converting the time-domain waveform into bipolar phase bits are:

1. Identify valid message locations from the bipolar phase bits data by correlating phase data with the Barker code.
2. Convert the valid message phase bits into symbol bits using the relationship of 10 carrier cycles per symbol.
3. Locate the Barker code in symbol data by checking the message synchronization character.
4. Compute and check the CRC of the message (a valid CRC is zero).
5. Compute the phase margin of the message
6. Repeat for the other five phase shifts (total of six possible phase shifts with six samples per cycle)
7. Repeat with a split-phase clipping level, effectively doubling the number of phase offsets checked.
8. Output the decoded code, start time, SNR, phase margin, and other information after converting decoded code into hexadecimal code.

As an example, the acquired waveform shown in Figure 3 is selected to demonstrate how the different components function in the decoding process. The most likely message locations are then computed by searching for windowed energy peaks (Figure 6). There is only one possible energy peak at sample number 9,798 with an energy number of 714 or a SNR of 12.9 dB, and the corresponding likely message start is sample number 7,938. All other energy peaks have SNRs lower than 0 dB. The most likely message is then extracted by including 1,800 samples prior to the most likely message start and 3,500 samples after the most likely message. The phase angle of the message [Figure 7(a)] is computed using a matched filter and converted to bipolar clipped phase [Figure 7(b)]. The clipped phase is then correlated with the Barker code to locate the Barker code. After the clipped phase bits are converted to symbol bits and the synchronization character is located, the binary value of the decoded message is then obtained: 0111 0010 0111 1010 1010 1100 1111 1101. The corresponding hexa-decimal code is identified as 727AACFD; 72 is the Barker code, 7AAC is the ID, and FD is the CRC. The letter G is added to indicate good CRC status, resulting in a final decode of G727AACFD with a time arrival of 0.3174 ms from the start of file time.

## 4. Performance

Two different experiments were used to evaluate the performance of the JSATS cabled system—one in a controlled laboratory environment and the second in near-dam field environments at the Bonneville Dam spillway and John Day Dam. This article briefly describes the decoding efficiency in the laboratory environment and at the Bonneville Dam spillway. Part 2 [22] describes in detail its performance at John Day Dam.

### 4.1. Performance in a Laboratory Environment

Performance tests were conducted in a tank lined with anechoic material [27]. To simulate range, a source level of 156 dB re μPa @ 1 m was used because it was close to the typical source level of existing JSATS transmitters [12]. The minimum source level of JSATS transmitters is 153 dB re μPa @ 1 m.

The encoded waveforms were transmitted at signal levels of 116, 106, 101, 96, 91, and 86 dB re 1 μPa @ 1 m (measured at the center frequency of 416.7 KHz), resulting in six levels of signal attenuation at −40, −50, −55, −60, −65, and −70 dB, respectively. Assuming the transmission loss is due only to spherical spreading, the six signal attenuation levels are equivalent to 100, 316, 562, 1,000, 1,778, and 3,162 m, respectively, in an ideal environment. A broadband spherical hydrophone (Model TC 4034, RESON, Slangerup, Denmark) was used to transmit the encoded signal. The cabled receiver was placed, hydrophone tip down, in the tank. Twenty-eight tag codes were used to represent the 14 different phase shift counts of all possible tag code combinations, with two tag codes randomly selected from each phase shift count category [27]. Decoding efficiency was calculated as the number of correctly decoded detections divided by the number of transmissions. A typical JSATS cabled Model 2008 hydrophone has a decoding efficiency of 59% at −55 dB; *i.e.*, a detection range of 562 m (decoding efficiency > 50%) in an ideal environment (Figure 8).

### 4.2. Performance in a Field Environment

Bonneville Dam spans the Columbia River between Oregon and Washington, approximately 234.3 km from the mouth of Columbia River and approximately 64 km east of Portland, OR. The spillway, constructed between 1933 and 1937, is usually acoustically the noisiest environment among the lower Columbia River dams.

In the field, the received waveform may be distorted by its passage through water, which in almost all cases is not homogeneous, and by multipath. Multipath distortion of a microtransmitter message is caused by the near simultaneous arrival at the hydrophone of two copies of a microtransmitter message that travel by different paths and differ in time of arrival by less than the transmit duration of the message. Most commonly, multipath results from an overlap in time at the receiver of a direct path and an indirect path message in which the indirect path message has been reflected off the water surface, bottom, or structures in the water. In all cases, the indirect path message lags the direct path signal. The message length in water is approximately 1.1 m; thus, an echo whose path length is less than 1.1 m longer than the direct path will overlap the direct path signal. If multipath signals do not overlap, they can result in more than one valid detection of a single transmission. For actual field deployment, individual hydrophones are usually baffled by plastic cones lined with an anechoic material to exclude loud noises emanating from structures downstream of the hydrophones. Baffling greatly increased the ratio of tag signals relative to background noise levels and significantly increased the percentage of successful tag decodes. For the performance results reported in this article, the hydrophones were not baffled.

The detection efficiency is defined as the number of detections divided by the number of transmissions. The transmitter was suspended in the water column at various distances from the receivers. The number of transmissions was estimated directly using the first and last detection time and the transmit interval of 1.04 s. If the transmitter was not decoded at the time expected, the original waveform would be reviewed manually to determine if it was a valid message. It would be counted as a detection if it was a valid message from the manual review. The detection efficiency was above 99.5% up to 107 m and 71.3% at 122 m.

Decoding efficiency was the number of valid decodes divided by the number of transmissions. If the time gap between decodes for the same tag code was less than 0.3 s (usually 0.001 to 0.005 s), then there was a multipath signal. Multipath decodes were subtracted from the raw total to compute the number of total valid decodes. One DSP + FPGA card was used to control two channels. The decoding efficiency was above 53% for channel 1 and 76% for channel 2 up to 107 m [Figure 9(a)].

Background noise was computed as the mean value of the cross-correlation values of rejected packets that did not meet the criteria of the JSATS detector. SNR was defined as the ratio of the peak cross-correlation value of a candidate message over the background noise. For a given environment, SNR is a function of detection range and decreases as range increases. At Bonneville Dam spillway, SNR started decreasing quickly after 50 m and was only approximately 4 at 122 m [Figure 9(b)].

## 5. Conclusions

The JSATS is a nonproprietary sensing technology developed by the U.S. Army Corps of Engineers, Portland District, for detecting and tracking small fish. Each cabled system is synchronized to a universal GPS clock, resulting in timing accuracy of 250 ns within a single system and 500 ns across multiple systems. The JSATS cabled system was evaluated extensively in both a controlled laboratory environment and a near-dam noisy field environment. The testing demonstrated the JSATS detection range of more than 500 m in an ideal laboratory environment. The system detection efficiency of 99.5% up to 107 m and average decoding efficiency of 64.5% resulted in a detection range greater than 107 m in the near-dam noisy field environment. The JSATS cabled systems have been deployed successfully on several major dams to acquire information for salmon protection and to develop more “fish-friendly” hydroelectric facilities.

## Figures and Tables

**Figure 1.** JSATS cabled system schematic showing main components and direction of signal acquisition and processing.

**Figure 2.** JSATS acoustic microtransmitter (Advanced Telemetry Systems, Inc., Isanti, MN, USA).

**Figure 3.** Typical microtransmitter BPSK signal consisting of 310 cycles and 1,860 samples: **(a)** complete waveform; **(b)** zoomed-in view for phase change demonstration.

**Figure 4.** JSATS cabled system components: **(a)** data collection array; **(b)** cabled hydrophone.

**Figure 5.** Correlation of an impulse noise that does not pass the JSATS detector: **(a)** wave; **(b)** cross-correlation.

**Figure 6.** Correlation of a candidate signal that passes the JSATS detector.

**Figure 7.** Phase angle around the most likely message, which is cycles 270 to 580 (310 total): **(a)** actual; **(b)** bipolar.

**Figure 8.** Decoding efficiency of a JSATS cabled hydrophone in an ideal environment.

**Figure 9.** Field performance results at Bonneville Dam spillway: **(a)** efficiency *vs.* range; **(b)** SNR *vs.* range.
